RETRACTED

# Genetic characterization of the highlander Tibetan population from Qinghai-Tibet Plateau revealed by X chromosomal STRs

**DOI:** 10.1371/journal.pone.0271769

**Published:** 2022-08-04

**Authors:** Xiao-na Li, Atif Adnan, Sibte Hadi, Wedad Saeed Al-Qahtani, Maha Abdullah Alwaili, Dalal S. Alshaya, Areej S. Jalal, Sayed A. M. Amer, Feng Jin

**Affiliations:** 1 School of Fundamental Sciences, China Medical University, Shenyang, Liaoning, P.R. China; 2 Department of Forensic Sciences, College of Criminal Justice, Naif Universsity of Security Sciences, Riyadh, Kingdom of Saudi Arabia; 3 Department of Biology, Collage of Sciences, Princess Nourah Bint Abdulrahman University, Riyadh, Saudi Arabia; 4 Department of Breast Surgery, The First Hospital of China Medical University, Shenyang, Liaoning, P.R. China; Xiamen University, CHINA

## Abstract

Tibetans are considered an East Asian ethnic group and primarily live in the high Tibetan plateau, the western Sichuan and Yunnan mountains of central and southern China, and areas throughout the Himalayas and around the Tibetan plateau. These people exhibit rare molecular machinery that allows them to adapt to hypoxic environments in the Qinghai-Tibet Plateau and make them a potential candidate for providing insights related to medical genetic, molecular medicine and human population studies. In the current study, we have genotyped 549 individuals with Investigator Argus X-12 Kit. For 12 X-STRs, a total of 174 unique alleles were found, among them DXS10134 and DXS10135 were the most polymorphic loci. All of the loci were in Hardy-Weinberg Equilibrium (HWE). The numbers of observed haplotypes in Highlander Tibetans males were 161,112, 96 and 108, respectively, whereas haplotype diversities (HD) were 0.9959, 0.9880, 0.9809 and 0.9873, respectively. The combined discrimination power for males (PDm) was 0.999 999 99701 and for females (PDf) was 0.999 999 999 999 9958. This study represents an extensive report on X chromosomal STR markers variation in the Highlander Tibetans population for forensic applications and population genetic studies.

## 1. Introduction

The enduring occupation of the Qinghai-Tibet Plateau, also known as the Himalayan Plateau, is one of the greatest mysteries for human beings [1]. The indigenous Tibetans have emerged from a series of adaptations to the ruthless environments [2–5]. Their ancient civilization was developed to the foundation of the Tibetan Empire which lasted from the 7th to 9th centuries AD. After the consolidation of the Qinghai-Tibet Plateau, the Tibetan Empire went through a series of wars to expand its territory [6]. During the reign of Tsenpo ("Emperor") Trisong Detsen (755–797 AD), the Tibetan Empire reached its zenith and ruled over western China and parts of Central Asia and South Asia. His armed forces even captured Chang’an, the capital of the Tang Empire, at 763 AD [7]. The historical and archaeological records indicated massive population migrations being involved in a series of military conquers [8], which could leave a profound legacy on the cultural and genetic diversity of human populations [9]. Tibetans, with a population size of 7.5 million, are settled in the Qinghai-Tibet Plateau and across China. When Tibet became an autonomous region of China in 1959, a large number of Tibetans migrated as refugees (approximately 1.5 million) to India, Pakistan, Bhutan, Nepal, and other countries. In last three decades, genetic studies particularly mtDNA analysis shed light on the material linages of Sino-Tibetan populations which showed that they have northern Asian origin because of northern Asian specific haplogroup A, D, G, and M8 [10, 11].

RETRACTED

Short tandem repeats (STRs) or microsatellites, are present in noncoding intron regions of the human genome and are extensively used for forensic identifications in forensic DNA laboratories all over the world [12–17]. STRs usually comprise of tandem repeat motif from 2–6 base pairs. STRs have more tendency to mutate as compared to single nucleotide polymorphisms (SNPs), which makes them a potential candidate for population studies, evaluation of human population biodiversity, and forensic applications. In forensic biology, when we obtain data using these STR markers, which are located on both autosomal and sex chromosomes, it can be served as a basic material for the characterization of genetic diversity between inter and intra-population [18–21]. Utilizations of X-chromosomal short tandem repeat (X-STR) have been fully established and characterize for kinship analysis and identification with specific reference to forensics [22]. X-STRs, which have the properties of both autosomal and uniparental genetic markers, are useful in testing the mother-son kinship [22–25]; sibling status of two females having the same biological father without reference to the father’s DNA; and grandmother/granddaughter relationships, as granddaughters theoretically carry at least one allele in common with the grandmother [26]. There are different X-STR multiplexes available for forensic cases and genetic studies [27–30]. But, the Investigator Argus X-12 Kit (QIAGEN, Hilden, Germany), which contains the amelogenin locus along with 12 X-chromosomal STR markers, has been used for worldwide populations. The genetic structure of Sino-Tibetan populations suggests the substantial involvement of the surrounding populations. Therefore, in this study, we have typed 549 individuals with X chromosomal STRs belongs to Sino-Tibetan. Moreover, we performed comprehensive population comparisons with reference populations that are closely related to cultural, geographical or linguistic groups to understand the genetic portray of the Tibetan population.

RETRACTED

## 2. Materials and methods

### 2.1. Population samples

To explore the genetic structure and forensic parameters of the Highlander Tibetan population from the Nagqu city in the north of the Tibet Autonomous Region (TAR) in China, blood samples were obtained on FTA cards from 549 volunteer donors (male = 249, female = 300) for X-STRs. All participants who were included in this study were unrelated individuals at least three generations. All participants gave their informed consent either orally and with thumbprint (in case they could not write) or in writing after the study aims and procedures were carefully explained to them. DNA isolation was performed using the ReliaPrep^TM^ Blood gDNA Miniprep System (Promega, Madison, USA.) according to the manufacturer’s instructions. A Nanodrop-2000 spectrophotometer (Thermo Fisher Scientific, Wilmington, DE, USA) was used to measure the DNA concentration and purity. Then DNA was diluted accordingly to make the final concentration 2 ng/ul and stored at −20°C until amplification.

### 2.2. Compliance with ethics guidelines

The study was approved by the ethical review board (2016–063) of the China Medical University, Shenyang, Liaoning Province, People’s Republic of China. All the experimental procedures were performed following the standards of the Declaration of Helsinki.

### 2.3. PCR amplification and STR typing

549 diluted DNA extracts and positive control samples (9947A, 9948) were amplified with Investigator Argus X-12 Kit, on a GeneAmp PCR System 9700 Thermal Cycler (Thermo Fisher Scientific, MA, USA) according to the manufacturer’s recommended protocol. After successful amplification, the PCR products were analyzed using an 8 capillary ABI 3500 DNA Genetic Analyzer with POP-4^TM^ polymer (Life Technologies) according to the manufacturer’s recommended protocol. GeneMapper Software version 4.0 (Life Technologies) was used for genotype assignment. DNA typing was performed according to the manufacturer’s recommended protocol using the locus panel and allele bins supplied by the manufacturers and allele designations corresponding with the allelic ladder supplied by the manufacturer. Genotyping nomenclature was based on the recommendations of the International Society for Forensic Genetics (ISFG) [31, 32].

### 2.4. Statistical analyses

Calculation of observed heterozygosity (*H*_O_), Hardy-Weinberg equilibrium (HWE) in and linkage disequilibrium (LD) were performed using Arlequin v3.5 [33]. Allele frequencies were calculated by counting the number of times each allele was observed and expressing as a fraction of the total. Fisher’s exact test was performed using an online tool (https://www.socscistatistics.com). The haplotype frequencies of four linkage groups (LG1, LG2, LG3, and LG4) [22, 34] were also computed by counting the number of times each haplotype was observed and haplotype diversity (HD) was calculated according to:

$$HD=\frac{n}{n-1}\left(1-\sum_{i}p_{i}^{2}\right)$$

where *n* is the male population size and *p*_*i*_ is the frequency of *i*th haplotype. Other forensic statistical parameters, such as the power of discrimination in females (PDF) and in males (PDM), the polymorphism information content (PIC), the power of exclusion (PE), the paternity index (PI) and the mean paternity exclusion chance (including MECKrüger, MECKishida, MECDesmarais and MECDesmarais Duo variants), were estimated using the online calculation tool available with the ChrX-STR.org 2.0 database [35].

RETRACTED

Population comparisons between the Highlander Tibetans population and 10 other Chinese reference populations [27, 36, 37] were performed. *F*_ST_ and corresponding *p* values for locus by locus comparisons were estimated using Arlequin v3.5 [33]. Nei’s genetic distances between Highlander Tibetans and sixteen reference populations [25, 38–47] were calculated using Philip 3.695 software [48] and a neighbor-joining tree was constructed using Mega 7.0 [49]. Reduced dimensionality spatial representation of the populations was performed using multi-dimensional scaling (MDS) with IBM SPSS Statistics for Windows, Version 23.0 (IBM Corp., Armonk, NY, USA). The STRUCTURE v.2.3.4 software [50] was used to calculate the ancestry component. The model-based analysis employed the length of the burnin period of 100,000 and Markov Chain Monte Carlo (MCMC) step of 100,000 under the ‘independent allele frequencies’ and ‘LOCPRIOR’ models with the k values ranging from 2 to 10 with 5 repeats each run.

## 3. Results and discussion

### 3.1. Allelic frequency and forensic parameter analysis for X-STRs

The 12 X-STRs were successfully amplified and genotyped. All of the loci were in Hardy-Weinberg Equilibrium (HWE) except for DXS10135 and DXS10134 in the female Highlander Tibetan population. However, when a sequential Bonferroni correction [51] was applied to mitigate against the so-called “multiple comparison problem” (where for a significance threshold *p*-value of 0.05, 5% of tests are likely to be significant by chance), no loci were found to be out of HWE (**S1 Table**). After the Exact Test, no significant difference was observed between male and female allele frequencies; therefore we pooled both together for calculating forensic parameters. These allelic frequencies and exact test along with p-values are documented in **S2A, S2B Table**. A total of 174 unique alleles were found at 12 X STR loci, among them DXS10134 and DXS10135 were the most polymorphic loci (each with 24 alleles) while DXS7423 was lest polymorphic locus (5 alleles). DXS10135 exhibited the highest forensic utility with a PIC of 0.902525, while DXS7423 had the lowest with a PIC of 0.441105. The combined power of exclusion (CPE) and the combined power of discrimination (CPD) for male and female were 0.9999906271, 0.99999999701, and 0.9999999999999958, respectively **(Fig 1)**. Mean exclusion chances (MEC Krüger, MEC Kishida, MEC Desmarais, and MEC Desmarais Duo) were 0.9999934, 0.999999986, 0.9999999864 and 0.9999978, respectively **(Table 1)**.

RETRACTED

**Fig 1:** Forensic parameters of the 12 X-STR loci in Highlander Tibetan population Parameters were calculated on the basis of allele frequencies in males (A), females (B) and both pooled together (C).

**Table 1:** Forensic parameters of the 12 X-STR loci in Tibetans population residing in Nagqu city in the north of the Tibet Autonomous Region (TAR) in China (n = 549).

	DXS10074	DXS10079	DXS10101	DXS10103	DXS10134	DXS10135	DXS10146	DXS10148	DXS7132	DXS7423	DXS8378	HPRTB
PIC	0.761191	0.742116	0.880687	0.69534	0.819545	0.902525	0.865624	0.891604	0.723229	0.441105	0.579435	0.636195
h	0.208844	0.224693	0.109702	0.263928	0.161114	0.090584	0.122201	0.099976	0.238541	0.47149	0.355942	0.308598
HET	0.791156	0.775307	0.890298	0.736072	0.838886	0.909416	0.877799	0.900024	0.761459	0.52851	0.644058	0.691402
PE	0.582729	0.554044	0.775646	0.486242	0.673081	0.814694	0.75033	0.795469	0.529574	0.213688	0.347114	0.415085
PD												
PD*f*	0.926419	0.916322	0.978354	0.88961	0.954702	0.984904	0.972892	0.981585	0.904869	0.690292	0.808682	0.84956
PD*m*	0.791156	0.775307	0.890298	0.736072	0.838886	0.909416	0.877799	0.900024	0.761459	0.52851	0.644058	0.691402
Mean paternity exclusion change												
MEC Krüger:	0.596465	0.567997	0.776259	0.511908	0.682136	0.81773	0.754058	0.797793	0.541492	0.250737	0.376603	0.433667
MEC Kishida:	0.761179	0.740369	0.87631	0.69534	0.819545	0.902525	0.865513	0.891277	0.723112	0.440982	0.579314	0.636195
MEC Desmarais:	0.761191	0.742116	0.880687	0.69534	0.819545	0.902525	0.865624	0.891604	0.723229	0.441105	0.579435	0.636195
MEC Desmarais Duo:	0.634571	0.610887	0.795969	0.556812	0.709632	0.829215	0.773348	0.812024	0.588006	0.303839	0.433097	0.490659

***PIC*:** Polymorphism information content; ***PE*:** Power of Exclusion; ***PD*:** Power of Discrimination ***HET*:** Heterozygotie; ***h***: Homozygotie

**PD*f*:** Power of Discrimination female; **PD*m*:** Power of Discrimination male

The above results are showing that the 12 X loci provide utility for forensic identification and paternity testing in the Highlander Tibetans in the Tibet province of China.

RETRACTED

### 3.2. Linkage disequilibrium (LD) analyses for X-STRs

Linkage disequilibrium refers to the non-random association of alleles at two or more loci and is sensitive indicator of the population genetic forces which assemble the genome. Nonrandom association of alleles and observed LD does not establish either there is linkage or a lack of equilibrium. It is important in human genetics and evolutionary biology because different factors can affect it and it can be affected by different factors. LD gives us the insight information about past events and it curbs the potential response to both natural and artificial selection. LD across the genome give us clues about the pattern of geographic subdivision, breeding system and population history, whereas disequilibrium in linkage among genomic region reflects the gene conversion, history of natural selection and mutation that cause gene-frequency evolution. How these factors affect LD between a particular pair of loci or in a genomic region depends on local recombination rates. LD tests were performed for all pairs of loci for the male population and twenty one pairs out of sixty six pairs showed LD. After applying a sequential Bonferroni correction [51], only eight pairs showed LD (DXS10101/DXS10103, DXS10074/DXS10103, DXS10146/DXS10134, DXS10101/DXS10134, DXS10148/DXS10074, HPRTB/DXS10101, DXS10146/DXS10135, DXS10146/DXS7423) **(S3A Table)**. For female pairs, twelve pairs showed LD after sequential Bonferroni correction (DXS10101/DXS10103, DXS10146/DXS8378, DXS10101/DXS8378, DXS10148/DXS10134, DXS10135/DXS10134, DXS10148/DXS10074, DXS10079/DXS10074, HPRTB/DXS10101, DXS10146/DXS10101, DXS10079/DXS10135, DXS10146/DXS7423, DXS10148/DXS10079) **(S3B Table).**

### 3.3. Haplotype analysis in males based on X-STRs

The 12 X-STR loci are clustered into four linkage groups according to their physical positions on the X chromosome [22, 34]: LG1 (Xp22) DXS8378-DXS10135-DXS10148, LG2 (Xq11) DXS7132-DXS10074-DXS10079, LG3 (Xq26) DXS10101-DXS10103-HPRTB and LG4 (Xq28) DXS7423-DXS10134-DXS10146. Each group of three markers is considered as one haplotype for the genotyping of males. These four haplotype groups (LG1, LG2, LG3, and LG4) showed a higher number of haplotypes in Highlander Tibetans males were 161,112, 96 and 108, respectively, whereas haplotype diversities (HD) were 0.9959, 0.9880, 0.9809 and 0.9873, respectively (**S4 Table**). In LG1, LG2, LG3, and LG4, the unique haplotypes were 101, 64, 55 and 56, respectively, while accepted heterozygosity was 0.8247, 0.7742, 0.7819 and 0.7400, respectively. Linkage disequilibrium refers to the non-random association of alleles at two or more loci in a population. When alleles are in linkage disequilibrium, haplotypes do not occur at the expected frequencies. We accepted to observe tight linkage between the STR trios in the four linkage groups and we would not assume any linkage among the STRs in different linkage groups. S3 Table demonstrated that these expectations were not been met. It is only DXS10101-DXS10103, HPRTB-DXS10101 in LG3 and DXS10146-DXS10134, DXS10146-DXS7423 in LG4. We also detected substantial LD among the groups: DXS10074 (LG2)-DXS10103 (LG3); DXS10101 (LG3)-DXS10134 (LG4); DXS10148 (LG1)-DXS10074 (LG2); DXS10146 (LG4)-DXS10135 (LG1). This might be the result of founder effects, mutations, random genetic drift, selection, and population admixture or stratification [52, 53]. Previous studies also suggested that recombination among linkage groups is not more than 50% [17, 54, 55]. Indeed, Diegoli *et al* [54] states against a simple model of independent X chromosomal linkage groups for these reasons.

RETRACTED

### 3.4. Inter-population differentiations

To compare the genetic relationship and population structure among Highlander Tibetans and other 10 Chinese populations, we have observed 80.1% of genetic variations (**Fig 2A**) via principal component analysis (PCA) on two components (PC1:53.3%, PC226.8%). Further, we have calculated pairwise Fst genetic distances and the Yi population from Liangshan showed closest (Fst = 0.00202) genetic distance while Kazakh population from Ily, Xinjiang showed (Fst = 0.0054) greatest genetic distance (**S5 Table**). Phylogenetic reconstruction (Neighbor-joining Tree) reveals two main clusters (**Fig 2B**), Kazakh and Uyghur population form the main cluster and other cluster was again subdivided into two clusters. Among these two sub-clusters, Tibetan, Yi, and Xibe populations are in one cluster while Han, Gelao, Manchu and Miao populations were in the second cluster. We also used these pairwise Fst genetic distances to generate heatmap and the result of the heat map is in accordance with the NJ tree (**S1 Fig**). The same population distribution patterns were observed in the MDS based on the pairwise Fst genetic distance (**Fig 2C**). Finally, the genetic makeup among the female samples was further investigated via hierarchical structure analysis (**Fig 2D**). We set k-values varying from 2 to 10 to get information of ancestry related to Highlander Tibetans and we have identified the best optimal predefined populations in seven (K = 7). We have observed consistent brown pink and blue common component among all populations. In Highlander Tibetans, we have observed 4 major components which are brown pink, blue and light green while a small portion of yellow and dark green. The only green component was present in Tibetans and Yi while the parrot green component was only present in Kazakhs and Uighurs. Green component was present in Highlander Tibetans while it was absent in Tibetans. One of the most difficult environmental stressors on human populations is altitude. Highlanders from Asia, America, and Africa have been shown to have a variety of biological adaptations [56–58]. Genetic and archaeological studies have documented a human presence on the plateau as early as 30,000 years before present (YBP) [59, 60]. Linguistic studies have suggested that the Tibetan and Chinese people share a common root ancestor and that the Tibetan-Chinese split took place ~6,000 YBP. A recent genetic study utilizing exome sequencing data estimated a divergence time of 2,750 years between Tibetans and Han Chinese [3]. Moreover, Nei’s genetic distance between Highlander Tibetans with 16 worldwide populations was computed which are summarized in **S6 Table**. Han population from Henan showed closest genetic distance (0.0152) followed by again Han population from northeast of China (0.0160) while West Croatian population showed greatest genetic distance (0.0995) among the studied population followed by Arab population from United Arab Emeritus (0.0942). We also performed PCA analysis (**Fig 3**) and observed 91.5% of genetic variations on two components (PC1:86%, PC2: 6.5%). To further explore the genetic homogeneity and heterozygosity, we subsequently performed MDS and reconstructed the N-J tree. In the MDS plot (**Fig 4**), the Chinese population formed a closed cluster on the left side except for the Kazakh population which placed on the lower middle of the plot, while other populations such as Serbian, Croatian and Arabs placed on right side of the plot. In the NJ tree (**Fig 5**), mainly two clusters were formed and Highlander Tibetan formed a cluster with the Southern Han population. The possible reason for this has been discussed in a linguistic study were the authors have suggested that the Tibetan and Chinese people share a common root ancestor and that the Tibetan-Chinese split took place ~6,000 YBP [ref]. A recent genetic study utilizing exome sequencing data estimated a divergence time of 2,750 years between Tibetans and Han Chinese [3]. The Kazak population clustered with Serbian, Croatian and Arabs. The same pattern was also observed in the heatmap (**S2 Fig**).

RETRACTED

**Fig 2:** Genetic structure and population relationship between Highlander Tibetan and other 10 populations; (A) Principal component analysis (PCA) revealed the genetic relationship on the basis of the first two components; (B) A two-dimensional scaling (MDS) plot of the Highlander Tibetan and other 10 populations; (C) A Neighbor-Joining tree explaining the phylogenetic relationship of Highlander Tibetan; (D) Genetic structure revealed by Structure from Highlander Tibetan female samples.

**Fig 3:** Principal component analysis (PCA) based on Nei’s genetic distance revealed by the first two components between Highlander Tibetans and 16 other populations.

**Fig 4:** A two-dimensional scaling (MDS) plot of the Highlander Tibetan and 16 other populations based on Nei’s genetic distances.

**Fig 5:** A neighbor-joining tree explaining the phylogenetic relationship of Highlander Tibetan and 16 other populations based on Nei’s genetic distances.

## 4. Conclusion

In the current study, we have typed 549 individuals with the Investigator Argus X-12 Kit (QIAGEN, Hilden, Germany). The genetic variation in the Highlander Tibetan population and its comparison to other relevant reference populations were analyzed using different statistical tests. These 12 X-STRs showed strong discrimination capacity, haplotype diversity, and random mating probability. These STRs could potentially be useful for regional or national reference reconstruction for forensic paternity testing, missing person investigations, and disaster victim identification. We have seen some additional green component in Highlander Tibetans in a hierarchical structure analysis and also observe some differences at the allelic frequency ranges between Highlander Tibetans and Tibetans.

## Supporting information

S1 Table Hardy–Weinberg equilibrium tests in the Highlander Tibetans female population residing in Nagqu city in the north of the Tibet Autonomous Region (TAR) in China (n = 549). A sequential Bonferroni correction was applied with a threshold p-value of 0.05.
(XLSX)

S2 Table A. Allele frequencies of the 12 X-STR loci in in the Highlander Tibetans population residing in Nagqu city in the north of the Tibet Autonomous Region (TAR) in China (n = 549). B. Fisher Exact test for population differentiation per locous between allelic frequencies of male and female sample in the Highlander Tibetans population residing in Nagqu city in the north of the Tibet Autonomous Region (TAR) in China (n = 549).
(XLSX)

S3 Table A. Linkage disequilibrium tests in the Highlander Tibetans female population residing in Nagqu city in the north of the Tibet Autonomous Region (TAR) in China (n = 300). A sequential Bonferroni correction was applied with a threshold p-value of 0.05. B. Linkage disequilibrium tests in the Highlander Tibetans male population residing in Nagqu city in the north of the Tibet Autonomous Region (TAR) in China (n = 249). A sequential Bonferroni correction was applied with a threshold p-value of 0.05.
(XLSX)

S4 Table Haplotype frequencies for the 4 linkage groups in the male Highlander Tibetan population residing in Nagqu city in the north of the Tibet Autonomous Region (TAR) in China (n = 249). (XLSX)

S5 Table Pairwise Fst genetic distances between Highlander Tibets and 10 other reference populations. (XLSX)

S6 Table Nei’s genetic distance between the Highlander Tibetans and and sixteen previously published populations based on twelve overlapping X-STR loci. (XLSX)

S1 Fig A heat map of pairwise Fst genetic distance values of the the Highlander Tibetan and other 10 populations. (JPG)

S2 Fig A heat map of pairwise Nei’s genetic distance values of the the Highlander Tibetan and other 16 populations. (JPG)
